# The Renshen Chishao Decoction Could Ameliorate the Acute Lung Injury but Could Not Reduce the Neutrophil Extracellular Traps Formation

**DOI:** 10.1155/2022/7784148

**Published:** 2022-08-29

**Authors:** Miao-En Yao, Yi Huang, Qing-Qing Dong, Yi Lu, Wei Chen

**Affiliations:** ^1^Longhua Hospital Shanghai University of Traditional Chinese Medicine, No. 725, South Wanping Road, Xuhui, Shanghai 200032, China; ^2^The Second Affiliated Hospital of Guangzhou University of Chinese Medicine, Guangzhou 510006, Guangdong, China; ^3^Department of Critical Care Medicine, Longhua Hospital Shanghai University of Traditional Chinese Medicine, No. 725, South Wanping Road, Xuhui, Shanghai 200032, China; ^4^Shanghai University of Traditional Chinese Medicine, 1200 Cai Lun Road, Zhangjiang Hi-TechPark, Pudong New Area, Shanghai 201203, China

## Abstract

The acute lung injury (ALI) causes severe pulmonary diseases, leading to a high mortality rate. The Renshen and Chishao have protective and anti-inflammatory effects against the ALI. To explore the protective effects of the Renshen Chishao (RC) decoction against the ALI, we established the lipopolysaccharide-indued ALI model and randomly divided the mice into seven groups: control group, ALI group, high-dose RC group, middle-dose RC group, low-dose RC group, middle-dose RC group + CXCR2 antagonist group, and ALI + CXCR2 antagonist group. We estimated the lung injury by the hematoxylin and eosin staining, the neutrophil extracellular traps (NETs) formations by the immunofluorescence colocalization and enzyme-linked immunosorbent assay (ELISA), and the CXCR2/CXCL2 pathway by the flow cytometry, ELISA, and real-time polymerase chain reaction. We conducted the high-throughput sequencing and enrichment analyses to explore the potential mechanisms. The results showed that the RC decoction pathologically ameliorated the lipopolysaccharide-induced lung injury and inflammatory response but failed to reduce the circulating and lung tissue NETs formation and the blood neutrophil percent. The high-dose RC decoction increased the plasma CXCL2 level, but the RC decoction had no effects on the neutrophilic CXCR2 levels. Under the inhibition of the CXCR2, the middle-dose RC decoction still decreased the lung injury score but as yet had unobvious influence on the NETs formation. Other potential mechanisms of the RC decoction against the ALI involved the pathways of ribosome and coronavirus disease 2019 (COVID-19); the target genes of inflammatory factors, such as *Ccl17, Cxcl17, Cd163, Cxcr5, and Il31ra*, and lncRNAs; and the regulations of the respiratory cilia. In conclusion, the RC decoction pathologically ameliorated the lipopolysaccharide-induced lung inflammatory injury via upregulating the CXCL2/CXCR2 pathway but could not reduce the circulating or lung tissue NETs formation.

## 1. Introduction

The acute lung injury (ALI) causes severe pulmonary inflammatory diseases, leading to a high mortality rate [1, 2]. The ALI pathogeneses included the disrupted pulmonary endothelium, alveolar epithelial injury, and dysregulated lung inflammation [2]. The excessive transepithelial neutrophil migration caused the hyperinflammatory response and lung vascular integrity loss [2–4]. Activated neutrophils released inflammatory factors such as protease, oxidant, leukotriene, and platelet-activating factor, resulting in the increased vascular permeability [4]. The neutrophil extracellular traps (NETs), released by the activated neutrophil, promoted the thrombosis formations and cytokine storm, leading to the extreme inflammatory response [5–7]. When the inflammatory response occurred in the lung, the neutrophil traveled to the lung by the chemotaxis of CXC chemokines including CXCL1, CXCL2, and CXCL5, combined with the CXCR2 receptor [8–10]. Interestingly, influenced by the circadian clock, the CXCL2/CXCR2 pathway disarmed the circulating neutrophils granule contents to reduce the pulmonary NETs-forming capacity and lung injury [11, 12].

The Renshen Chishao (RC) decoction includes the herbs of Renshen and Chishao, which ameliorated the lung injury or inflammatory diseases. In the *Staphylococcus aureus*-induced ALI mice model, the ginsenoside Rb1, a herb Renshen extract, alleviated the apoptosis and oxidative damage through the death receptor-mediated and endoplasmic reticulum stress-mediated pathways [13]. In the lipopolysaccharide- (LPS-) induced ALI mice model, administration of panaxydol, the Renshen active ingredient, decreased the inflammation severity, lung edema, and pathological changes, via the Keap1-Nrf2/HO-1 pathway upregulation [14]. The Xuebijing injection, which contains the compound in Chishao, reduced the cecal ligation and puncture-induced lung permeability, by upregulating the TOLLIP expression [15]. In the rat cholestasis model, the Chishao ameliorated the disease severity and inflammatory response by inhibiting the nuclear factor-*κ*B-NLRP3 inflammasome pathway [16].

Although previous studies have reported the Renshen or Chishao single effect, the RC decoction integrated effect against the ALI was as yet unclear. Therefore, we explored whether the RC decoction could ameliorate the ALI and inhibit the NETs formation in a LPS-induced ALI mice model. Through the high-throughput sequencing and enrichment analyses, we found potential mechanisms of the RC decoction against the ALI and chose the CXCL2/CXCR2 pathway to verify.

## 2. Methods and Materials

### 2.1. The RC Decoction Preparation

The RC decoction, containing Renshen (ginseng: the dry root of *Panax Ginseng C. A. Mey.*) and Chishao (red peony root: the root of *Radix Paeoniae Rubra*), was purchased from the LongHua Hospital Shanghai University of Traditional Chinese Medicine. Weighing 48.26 g for both, the herbs were soaked for 1 h in 775 ml double distilled water, decocted for 1 h and 25 min, and obtained 148 ml liquid after filtering. Adding 575 ml water again, the herbs were decocted for 1 h and 25 min to obtain 102 ml liquid. The liquids obtained for two times (148 ml and 102 ml) were mixed and stored at −40°C for 8 d to a thick paste. We put the thick paste in the vacuum freezer dryer (LGJ-10D, BEIJING SIHUAN Technology Co. Ltd, Beijing, China) at −60°C for three days. We pounded the dried thick paste into the freeze-dried powder (28.52 g), storing it at −20°C protected from light.

We searched the RC decoction active compounds from the traditional Chinese medicine database and analysis platform (TCMSP) database (https://tcmsp-e.com) and screened the ingredients with drug-likeness (DL) ≥ 0.18 and oral availability (OB) ≥ 30% (Table 1).

### 2.2. Animal Experiment

A total of 63 male Balb/c mice (23–30 g), purchased from the Shanghai Lingchang Biological Technology Co., Ltd (Shanghai, China), were maintained in the 23–27°C standard environment with 12-hour light/12-hour dark cycle. This experiment was approved by the LongHua Hospital Shanghai University of Traditional Chinese Medicine Ethics Committee (certification number: LHERAW-20018).

We established the LPS-induced ALI model according to the protocol [17]. After anesthesia (1% sodium pentobarbital, 60 mg/kg, intraperitoneal [i.p.] injection), we used a cotton to suspend the mice on a board through its front incisors. We pulled the tongue forward and instilled 53 ± 6 *μ*L phosphate buffer saline (PBS) dissolved with LPS (3 mg/kg, cat. No: L2880; Sigma-Aldrich, St Louis, MO, USA) into the posterior oropharynx. To make the reagent spread over the whole lung, we rotated the mice towards the right, left, forward, and backward within 1 min. We intragastrically gave the saline or the RC decoction to the mice at about two, 24, and 48 h after the ALI challenge.

For the antagonist groups, the mice received CXCR2 antagonist (SB 225002, 3 mg/kg/d, i.p. Injection, cat. No: S7651, Selleckchem, Houston, USA) once per day from the day before the ALI challenge to two days after the ALI challenge (four days in total).

In order to balance the inflammation levels differences among groups caused by the circadian clock [11, 12], we gave the interventions to the mice with the same sequence in different groups in the same time periods.  Figure 1 showed the flowchart and groups.

Euthanized at 60 h after ALI (1% sodium pentobarbital [45–60 mg/kg], intraperitoneal [i.p.] injection), we collected the blood via the cardiac puncture, leading to the sacrifice of the mice eventually. For flow cytometry, we stored about 200 *μ*L blood sample into an EDTA anticoagulant tube. The remaining blood samples were stored in the citric acid anticoagulant tube for the plasma isolation (3000 rpm, 10 min, 20°C; stored at −80°C) and neutrophil extraction (mixing up two or three blood sample; using density gradient centrifugation according to the mice peripheral blood neutrophils isolated kit, TIAN JIN HAO YANG Biological Manufacture CO., Ltd., Tianjin, China). The left lung was collected for weighing the wet weight, and the right lower lung for examining the histopathological changes.

### 2.3. H&E Staining and Lung Injury Scoring System

We harvested the right lower lung tissues to fix in the 4% paraformaldehyde and embedded them in the paraffin for the hematoxylin and eosin (H&E) staining. Via an inverted fluorescence microscope (Nikon Ti–U, Japan), images of the lung tissues cross sections were obtained at 20 different high-power fields (400x magnification). We measured the inflammation and injury degrees according to the lung injury scoring system [18], the neutrophils, airspaces proteinaceous debris, and hyaline membranes amounts, and the alveolar septum thickness were estimated.

### 2.4. Lung Immunofluorescence

The deparaffinized and rehydrated slices of right lower lung sections dealt with antigen retrieval and blocking. We incubated the slices overnight at 4°C with the first antibody against cit-H3 diluted 1 : 1000 (cat. No: ab5103, Abcam). Then, we incubated the slices with the horseradish peroxidase- (HRP-) conjugated second antibody, followed by the CY3-conjugated tyrosinase fluorescent probe (cat. No: SD0159, Shanghai Siding Biological Technology Co., Ltd, China). We washed the slices via the tris buffered saline tween and heat-treated them via the microwave oven. Repeating the previous steps, we incubated the slices with the first antibody against MPO diluted 1 : 100 (cat. No: ab208670, Abcam) and the HRP-conjugated second antibody, followed by the 488-conjugated tyrosinase fluorescent probe (SD0159, Shanghai Siding Biological Technology Co., Ltd, China). Subsequently, we stained the slices with DAPI, scanned them using the 3Dhistech Pannoramic MIDI (Hungary), and measured them via the CaseViewer 2.4. Using the ImageJ 1.53j “colocalization” plugin, the NETs formation was detected by the MPO (green), DAPI (blue), and cit-H3 (red) immunofluorescence colocalization analyses.

### 2.5. Enzyme-Linked Immunosorbent Assay

We measured the plasma chemokines CXCL2 concentration using the ELISA kit (cat. No: SDM0083, Shanghai Siding Biological Technology Co., Ltd, China) according to the manufacturer's instructions. Then, we detected the absorbances at 450 nm via the Infinite F50 microplate reader (TECAN, Switzerland).

We measured the plasma neutrophil elastase- (NE-) DNA complexes to detect the circulating NETs, using a Sandwich ELISA [19, 20]. Overnight, the 96-well microtiter plates (cat. No: 44-2404-21, Thermo Scientific, Waltham, MA) were coated by the capture antibody against NE (cat. No: ab68672, abcam; 50 *μ*L/well, 4°C) diluted in the carbonate-bicarbonate buffer (PH 9.6, cat. No: C3041, Sigma-Aldrich, St Louis, MO; 1 : 1000). After the blocking (5% bovine serum albumin, 200 *μ*L/well), we added the plasma sample (50 *μ*L/well; adding healthy volunteer plasma for the positive control) and incubated the peroxidase-conjugated detection antibody against DNA (cat. No: 11774425001, Cell Death Detection ELISA^plus^ Kit, Roche). We measured the optical density (OD) at 405 nm and 490 nm by the Synergy H1MF microplate reader (BioTek, USA). Finally, we got the OD_405–490_ index by dividing the sample OD_405–490_ values by the positive control OD_405–490_ values.

### 2.6. Flow Cytometry

We stained the whole blood sample (EDTA anticoagulant) with the CD11b-FITC (anti-mouse, cat. No: 11-0112-82, Thermo Scientific), Ly6G-APC (anti-mouse, cat. No: 127614, Biolegend), and CXCR2-PerCP/Cyanine5.5 (anti-mouse, cat. No: 149308, Biolegend) antibodies. The cells percent (neutrophil: Ly6G + CD11b; CXCR2^+^ neutrophil: Ly6G + CD11b + CXCR2) was measured by the flow cytometer (Celesta, BD, USA) and analyzed by the Flowjo 10.7.

### 2.7. Real Time PCR Analysis

Using the real-time reverse transcription-polymerase chain reaction (RT-PCR), we detected the *Cxcr2* and *Cxcl2* relative mRNA levels of the neutrophil (isolated from the whole blood). We extracted the total RNA via RNA extracting column (cat. No: B0004DP, EZBioscience), generated the cDNA through reverse transcription conducting (cat. No: A0010CGQ, EZBioscience), and amplified the cDNA by SYBR dye, Taq DNA polymerase, and ROX2 (cat. No: A0012-R2, EZBioscience). The gene primers adding to the reaction system were as follows: *Cxcr2* (forward: 5′-GCTCAC AAACAG CGTCGTAG-3′; reverse: 5′-ACCAAG GAGTTC CCCACAAG-3′), *Cxcl2* (forward: 5′-CCAGAC AGAAGT CATAGCCACT-3′; reverse: 5′-GGCACA TCAGGT ACGATCCA-3′), and *β-actin* (forward: 5′-CCTGTA CGCCAA CACAGTGC-3′; reverse: 5′-ATACTC CTGCTT GCTGATCC-3′). We conducted the cycling program by the Applied Biosystems 7500 Real-Time System (Thermo Fisher Scientific Inc., USA): 95°C, 5 min; 40 cycles, 95°C, 10 s; 58°C, 15 s; 72°C, 30 s, using the 2^−△△Ct^ method to calculate the relative mRNA levels (normalize to *β-actin*).

### 2.8. High-Throughput Sequencing

We used the TRIzol® Reagent (Invitrogen, USA) to extract the lung tissue samples total RNA (the control group [*n* = 3], ALI group [*n* = 3], and MRC group [*n* = 3]). The RNA quality was examined through the 2100 Bioanalyser (Agilent, USA), and the RNA concentration was quantified by the ND-2000 (NanoDrop Technologies, USA). Using 1 *μ*g total RNA, we constructed the cDNA library by the TruSeqTM RNA sample preparation Kit (Illumina, USA). The cDNA library was purified, selected for 300 bp fragments, and amplified by 15 PCR cycles (Phusion DNA polymerase, New England Biolabs, USA). We sequenced the library by the Illumina HiSeq xten/NovaSeq 6000 sequencer (Illumina, USA), with the reads length of 150 bp.

After the trim and quality control (SeqPrep: https://github.com/jstjohn/SeqPrep and Sickle: https://github.com/najoshi/sickle), we aligned the clean reads (HISAT2: https://ccb.jhu.edu/software/hisat2/index.shtml) to the reference genome (https://asia.ensembl.org/Mus_musculus/Info/Index) using orientation mode [21]. We assembled the sample mapped reads through the StringTie (https://ccb.jhu.edu/software/stringtie/index.shtml?t=example) [22]. We quantified the gene abundances by the RSEM (https://deweylab.biostat.wisc.edu/rsem/) and calculated the transcript expression levels with the transcripts per million reads (TPM) method [23]. Using the EdgeR, the differential expressed genes were identified with the *P*-value<0.05 and |log2FC|>1 [24], present in the cluster heatmap via the ClustVis (https://biit.cs.ut.ee/clustvis/).

### 2.9. Enrichment Analyses

By the “org.Mm.eg.db,” “DOSE,” “enrichplot,” and “clusterProfiler” (https://www.bioconductor.org) R packages, for the differential expressed genes, we conducted the gene ontology (GO) enrichment analyses including biological process (BP), cellular component (C-C), and molecular function (MF), and the KEGG signal pathway enrichment analysis. We chose the CC, MF, BP, and KEGG pathways with *P* value < 0.05. The CC, MF, and BP with top 10 significant *P* values were shown in the bar graphs, and the KEGG pathways with top 20 enriched gene ratios in the dot graph.

### 2.10. Statistical Analysis

We used Stata/MP 16.0 software for statistical analyses and expressed quantitative data as mean ± standard deviation (SD) or median (interquartile range). Student's *t*-test, Wilcoxon rank-sum test, and one-way analysis of variance (ANOVA) were used. *P* value < 0.05 was considered as statistical significance.

## 3. Results

### 3.1. The RC Decoction Effects against the ALI

After being treated with the HRC, MRC, or LRC, the lung swelling, congestion, and hyperemia were alleviated, but without dose-dependence. The lung wet weight/body weight ratios (LW/BW) were increased (Figure 2(a), *P* < 0.0001) by the ALI challenge and decreased by the HRC treatment (Figure 2(a), *P*= 0.0333). The MRC (*P*=0.5379) and LRC (*P*=0.3125) could not obviously decrease the LW/BW (Figure 2(a)). These results indicated that the HRC, MRC, and LRC ameliorated LPS-induced lung injury in vivo, and the HRC more efficaciously inhibited the lung edema.

As shown in the HE staining, challenged by the ALI, more alveolar and interstitial space neutrophil amounts, thicker alveolar wall, and more hyaline membrane amounts existed (Figure 2(b)). Treated by the HRC, MRC, and LRC, the lung inflammatory damage levels decreased (Figure 2(b)). Quantified by the histologic lung injury scores, the HRC, MRC, and LRC groups decreased the lung injury compared with the ALI group (Figure 2(b); *P* < 0.0001,*P*=0.0004, *P*=0.0012). The HRC and MRC groups had lower scores than the LRC group (*P*=0.013,*P*=0.013). The difference in scores between the HRC and MRC groups was insignificant (*P*=1.000). Taken together, the RC decoction reduced pulmonary inflammatory injuries, and the HRC and MRC had stronger effects than the LRC.

### 3.2. The RC Decoction Effects on the Neutrophil Extracellular Traps

The circulating NE-DNA OD_405-490_ index was significantly increased in the ALI group compared with the control group (Figure 3(a), *P*=0.0268). Compared with the ALI group, the HRC, MRC, and LRC groups upregulated the OD_405-490_ index without statistical significance (*P*=0.2963,*P*=0.0770,*P*=0.7494). The results showed that the RC decoction had unobvious effects on the circulating NETs levels.

The lung tissue immunofluorescence image in the control group showed that the small amount green stain (myeloperoxidase) surrounded the blue stain (nucleus), while, in the ALI group, it showed that the brightness red, green, and blue stains partially overlapped. The HRC, MRC, and LRC groups slightly decreased the stains intensities (Figure 3(b)).

For quantitative analyses, the DAPI and MPO and cit-H3 synthetic mean fluorescence intensities (MFI) were higher in the ALI group than the control group (Figure 3(b), *P*=0.0016 and *P*=0.0233). Although the HRC and MRC groups suppressed the NETs levels to some extent, the MFI differences between the RC groups and ALI group were insignificant (Figure 3(b)). Hence, the RC decoction failed to reduce the pulmonary NETs accumulation.

### 3.3. Potential Mechanisms of the RC Decoction against the ALI

The high-throughput sequencing showed that the 194 genes expressions increased after the ALI and decreased after the MRC intervention, while the 99 genes expressions manifested an opposite trend. In total, 293 genes were selected to conduct the GO and KEGG enrichment analyses. The RC decoction potentially alleviated the ALI through the respiratory cilium assembly/movement and cell organelle assembly/movement in the BPs (Figure 4(a)); the cytoplasm, ribosome, and axoneme in the CCs (Figure 4(b)); and the ribosome structural constituent in the MF (Figure 4(c)). The RC decoction also regulated the ribosome and coronavirus disease 2019 (COVID-19) KEGG pathways.

We selected 40 genes with top 20 |log2FC| values (ALI group vs. MRC group) to generate the cluster heatmap (Figure 5). The RC decoction targeted the inflammatory and immune factors genes, such as interleukin 31 receptor A (*Il31ra*), CD5 antigen-like (Cd5l), and Immunoglobulin kappa variables; and the long noncoding RNAs (lncRNA) genes, such as Gm20463, Gm15832, and Gm47882.

### 3.4. Inflammatory Factors Involved in the RC Decoction Effects

As shown in Figure 6, compared with the ALI group, the chemokine (C–C motif) ligand 17 (*Ccl17*), V-set and immunoglobulin domain containing 1 (*Vsig1*), chemokine (C-X-C motif) ligand 17 (*Cxcl17*), and chemokine (C-X-C motif) ligand 2 (*Cxcl2*) TPMs decreased after the RC decoction intervention (|log2FC| = 1.91, 1.89, 1.20, 0.98; *P*=0.034, 0.042, 0.004, 0.015), while the CD163 antigen (*Cd163*), CD5 antigen-like (*Cd5l*), CD79A antigen (*Cd79a*), chemokine (C-X-C motif) receptor 2 (*Cxcr2*), chemokine (C-X-C motif) receptor 5 (*Cxcr5*), and interleukin 31 receptor A (*Il31ra*) TPMs increased (|log2FC| = 1.51, 3.66, 1.20, 1.47, 1.50, 2.73; *P*=0.001*P*=0.001, 0.031, 0.009, 0.003, 0.021, 0.004). Subsequently, we selected the *CXCL2/CXCR2* pathway to verify.

### 3.5. The RC Decoction Effects on the Neutrophilic CXCL2/CXCR2 Pathway

The flow cytometry in the Figure 7(a) revealed that the ALI challenge significantly increased the neutrophil percent and the neutrophil surface CXCR2 expression (*P*=0.0016, *P*=0.0023), but the HRC, MRC, and LRC treatments had insignificant effects on them. According to the ELISA, the plasma CXCL2 levels were suppressed by the ALI group (Figure 7(b), *P*=0.0326), elevated by the HRC group (*P*=0.0460), and unchanged by the MRC and LRC groups (*P*=0.3672, *P*=0.0805).

Consistent with the CXCR2 protein level, the *Cxcr2* relative mRNA level was increased after the ALI challenge (Figure 7(c), *P*=0.0339); and inconsistent with the CXCL2 protein level, the *Cxcl2* relative mRNA expression was activated by the ALI challenge (Figure 7(d), *P*=0.0310). The HRC, MRC, and LRC treatments failed to regulate the *Cxcr2* and *Cxcl2* relative mRNA levels.

Collectively, the RC groups had insignificant effects on the neutrophil percent and neutrophilic CXCR2 expression, but the HRC increased the circulating CXCL2 level to promote the combination of the CXCL2 and CXCR2. Hence, the RC decoction ameliorated the lung injury through the CXCR2/CXCL2 pathway activation.

### 3.6. The CXCR2 Antagonist SB 225002 Suppressed the CXCR2 Expression

The CXCR2 antagonist SB 225002 was used to confirm the RC decoction effects against the ALI when suppressing the CXCR2/CXCL2 pathway.

Compared with the MRC group, the MRC + antagonist group downregulated the CXCR2 expression at both the protein and mRNA levels (Figures 8(a) and 8(b), *P*=0.0229 and *P*=0.0092) but could not regulate the CXCL2 expression (Figures 8(c) and 8(d)). Compared with the ALI + antagonist group, the *Cxcl2* mRNA level was suppressed in the MRC + antagonist group (Figure 8(d), *P*=0.0035).

Taken together, the CXCR2 antagonist SB 225002 suppressed the CXCR2 expression at both the protein and mRNA levels.

### 3.7. The RC Decoction Effects under the CXCR2 Expression Suppression

The lung surface swelling, congestion, and hyperemia and the LW/BW were similar between the MRC + antagonist and ALI + antagonist groups (Figure 9(a)). The lung injury score was lower in the MRC + antagonist group than the ALI + antagonist group (Figure 9(b), *P*=0.0203). The results suggested that the RC decoction reduced the lung injury through other pathways besides the CXCR2/CXCL2.

Different from the result (Figure 7(a)) without the CXCR2 expression suppression, the MRC increased the circulating neutrophil percent (Figure 9(c), *P*=0.0419). Similar to the result without the CXCR2 expression suppression, the differences in the circulating NE-DNA level and pulmonary NETs amount were unobvious between the MRC + antagonist and ALI + antagonist groups (Figures 9(d) and 9(e)). The outcomes indicated that, under the CXCR2/CXCL2 pathway inhibition, the RC decoction as yet had insignificant effects on the NETs formation but increased the circulating neutrophil level.

## 4. Discussion

In this study, we administrated the LPS-induced ALI mice with the RC decoctions. The major findings were described as follows. The RC decoction ameliorated the LPS-induced lung inflammatory injury but failed to reduce the circulating and lung tissue NETs formation. For the potential mechanisms, the RC decoction was involved in the respiratory cilium assembly/movement and the ribosome structural constituent, as well as the ribosome and COVID-19 KEGG pathways. The RC decoction might target the inflammatory factors genes, such as *Ccl17*, *Cxcl17*, *Cd163*, *Cxcr2*, *Cxcr5*, *Cxcl2*, and *Il31ra*, and the lncRNAs genes. For the verification, the RC decoction reduced the lung injury through the pathways besides the CXCR2/CXCL2.

According to the previous studies, the Renshen and Chishao, two herbs of the RC decoction, reduced the lung injury, inflammatory response, and neutrophil activity. The Renshen had anti-inflammation effects through the neutrophil activity inhibition. The red-ginseng-derived compound, ginsenoside Rg3, reduced the neutrophil migration in the chronic obstructive pulmonary disease exacerbation murine model by downregulating the neutrophils PI3K activities [25]. The ginsenoside Rg6 suppressed the neutrophil infiltration and the tumor necrosis factor-*α* (TNF-*α*) expression in the lung tissue to promote the recovery from the LPS-induced lung damages [26]. Other experiments also showed the protective effects of Renshen against the ALI via the inflammatory factor regulation. In the ALI rat model, the ginsenoside Rb1 attenuated lung injury through the inflammatory factors inhibition such as interleukin (IL)-8, TNF-*α*, and MCP-1 [27]. In another ALI mice model, via the mammalian target of rapamycin-related pathway, the ginsenoside Rg3 suppressed the proinflammatory mediators such as TNF-*α*, IL-1*β*, and IL-6 and promoted the anti-inflammatory mediators such as IL-10 and transforming growth factor-*β* [28].

Few studies reported the Chishao anti-inflammatory effects against the ALI [16]. The Xuebijing injection, containing the Chishao ingredient, had therapeutical effects against the inflammatory diseases in clinic. In the randomized double-blinded trial with 60 severe COVID-19 patients, the Xuebijing injection suppressed the cytokine storm by regulating the TNF-*α*, IL-6, and IL-8 [29]. For 50 patients undergoing cardiopulmonary bypass surgery, the Xuebijing injection reduced the atelectasis incidence, increased the PaO2/FiO2 ratio, via downregulating the inflammatory mediator, suppressing the neutrophil infiltration, and upregulating the IL-10 levels [30]. A meta-analysis including 17 randomized controlled trials suggested that the Xuebijing injection combining with the ulinastatin for the sepsis patients decreased 28-day death, shortened mechanical ventilation duration, lowered procalcitonin levels, and reduced C-reactive protein concentrations [31].

The differential expressed genes GO analyses indicated that the RC decoction potentially regulated the respiratory cilia and ribosome functions. The respiratory cilia were the innate defense to clear the inhaled pathogens from the lung [32]. Targeted by the bacteria, viruses, or fungi, the impaired cilia disrupted the mucociliary clearance and worsened the infection [32]. At the COVID-19 infection onset, ciliated cells were the major target [33], resulting in the cilia shrinking, cilia loss, and ciliary beating reduction [34, 35]. In our study, the RC decoction might improve the cilia movement and assembly, promoting the pathogens clearance and alleviating the lung injury. In the public single-cell RNA sequencing datasets bioinformatic analysis, the ribosome downregulation in lung tissue decreased the COVID-19 severity [36]. And our study indicated that the RC decoction involved in the ribosome pathway, so we inferred that it might treat the COVID-19 by regulating the ribosome.

In this study, several inflammatory factors were the potential RC decoction target genes against the ALI, consistent with the previous experiments results [37, 38]. The ginsenoside Rg5 : Rk1 reduced the TNF-*α*/interferon-*γ*-induced elevated CCL17 expression in the keratinocytes [37]. Treating the colitis mice with the ginsenoside Rg1 and Rock1 inhibitor Y27632 upregulated the peripheral blood CD11b^+^*F*4/80^+^CD163^+^ M2 macrophages [38]. Our result showed that the lncRNAs, participating in the pulmonary inflammation and apoptosis [39, 40], were also the RC decoction target genes. The Renshen was reported to regulate the lncRNA levels: the ginsenoside Rb3 increased the lncRNA H19 level and alleviated the smoke-induced lung injury [41].

As the CXCR2/CXCL2 pathway involved in the inflammatory response [8–10], we chose it for the mechanism verification, although the *Cxcl2* |log2FC| was less than 1 (0.98). The HRC increased the plasma CXCL2 levels and decreased the lung inflammatory injury but failed to reduce the blood neutrophil percent and the NETs formation. This result could be interpreted with the CXCR2/CXCL2 pathway dual effects on neutrophils: the chemotaxis [8–10] and the disarming effects [11, 12]. The MRC elevated effects on the CXCL2 levels lessened the neutrophils capacity to generate the NETs but exacerbated the neutrophils chemotaxis from bone marrow to blood and lung. So, the synthetic effects manifested as unobvious influence on the NETs levels, but the disarming effects on the neutrophil reduced the lung injury.

Interestingly, under the CXCR2 expression suppression, the MRC upregulated the circulating neutrophil percent. We inferred that reducing the neutrophils chemotaxis to the lung might cumulate the circulating neutrophils, and the CXCR2 might antagonize the RC decoction elevated effects on the neutrophil percent. After suppressing the CXCR2, the RC decoction still pathologically ameliorated the lung injury, so we deduced that the RC decoction relieved the lung inflammatory damage through other pathways besides the CXCR2/CXCL2.

We firstly explored the *Panax Ginseng C. A. Mey.* and *Radix Paeoniae Rubra* effects on the lung injury and NETs formation in the LPS-induced ALI mice model. The results indicated the RC decoction possible clinical values against the lung inflammatory injury and eliminated its therapeutical effect on the NETs excessive formation. We gave the intervention in a method to avoid the circadian clock relevant bias (Figure 1) [11, 12].

The neutrophil purity for the RT-PCR was insufficient (approximately 31% tested by the flow cytometry: Ly6G + CD11b). Nevertheless, as shown in the Bgee database (https://bgee.org), the mice *Cxcr2* and *Cxcl2* circulating mRNA were mainly expressed on the granulocyte (expression score: 99.56, 99.36), so the RT-PCR results primarily presented the neutrophil mRNA levels, solving the limitation to some extent.

## 5. Conclusions

The RC decoction pathologically ameliorated the LPS-induced lung inflammatory injury via upregulating the CXCL2/CXCR2 pathway but failed to reduce the circulating and lung tissues NETs formation, and the blood neutrophil percent. Other potential mechanisms involved the ribosome and COVID-19 pathways; the inflammatory factors genes, such as *Ccl17, Cxcl17, Cd163, Cxcr5, and Il31ra*, and the lncRNAs genes; and the respiratory cilia functions.

## Figures and Tables

**Figure 1:** Flowchart of the experiment. We built the LPS-induced ALI model, gave the drugs (two, 24 and 48 h after ALI), and conducted the sacrifice (60 h after ALI) for the mice with the same sequence in different groups in the same time periods. We randomly divided the mice into seven groups: (1) control group (*n* = 10, untreated); (2) ALI group (*n* = 10, ALI model + saline [0.1 ml/10 g/d]); (3) HRC group (*n* = 10, ALI model + high-dose RC decoction [2318 mg/kg/d]); (4) MRC group (*n* = 10, ALI model + middle-dose RC decoction [1159 mg/kg/d]); (5) LRC group (*n* = 10, ALI model + low-dose RC decoction [580 mg/kg/d]); (6) MRC + antagonist group (*n* = 10, ALI model + middle-dose RC decoction + CXCR2 antagonist); (7) ALI + antagonist group (*n* = 3, ALI model + CXCR2 antagonist).

**Figure 2:** The RC decoction effects against the ALI. (a) Lung wet weight/body weight ratio (LW/BW). (b) Lung HE staining (200x magnification, bar = 50 *μ*m) and injury scores. Data is presented as mean ± SD; ^*∗∗*^*P* < 0.01, ^*∗*^*P* < 0.05.

**Figure 3:** The RC decoction effects on the neutrophil extracellular traps (NETs). (a) Plasma NE-DNA relative concentration (ELISA). (b) Lung tissues NETs formations detected by the immunofluorescence (left, bar = 50 *μ*m; red: cit-H3, green: myeloperoxidase, blue: DNA), with the colocalization quantitative analyses (right). Data is presented as mean ± SD or median (interquartile range); ^*∗∗*^*P* < 0.01, ^*∗*^*P* < 0.05.

**Figure 4:** The differential expressed genes GO enrichment analyses after the MRC intervention. (a) Biological processes with top 10 significant *P* value. (b) Cellular components with top 10 significant *P* value. (c) Molecular functions.

**Figure 5:** The RC decoction target genes cluster heatmap against the ALI. The genes with the top 20 |log2FC| values (ALI group vs. MRC group) in the upregulated and downregulated RC decoction target genes against the ALI.

**Figure 6:** The inflammatory factors involved in the RC decoction effects against the ALI. The gene transcripts per million reads (TPM) comparisons among the control group, ALI group, and MRC group. Data is presented as mean ± SD; ^*∗∗*^*P* < 0.01, ^*∗*^*P* < 0.05.

**Figure 7:** The RC decoction effects on the neutrophilic CXCL2/CXCR2 pathway. (a) The blood neutrophil (NEU) and CXCR2^+^ NEU (flow cytometry) percent. (b) Plasma CXCL2 concentration (ELISA). (c) The neutrophilic *Cxcr2* gene relative mRNA expression (RT-PCR, normalized to *β-actin*). (d) The neutrophilic *Cxcl2* gene relative mRNA expression (RT-PCR, normalized to *β-actin*). Data is presented as mean ± SD or median (interquartile range); ^*∗∗*^*P* < 0.01 and ^*∗*^*P* < 0.05.

**Figure 8:** The CXCR2 antagonist SB 225002 suppressed the CXCR2 expression. (a) The blood CXCR2^+^ neutrophil (NEU) percent (flow cytometry). (b) The neutrophilic *Cxcr2* gene relative mRNA expression (RT-PCR, normalized to *β-actin*). (c) Plasma CXCL2 concentration (ELISA). (d) The neutrophilic *Cxcl2* gene relative mRNA expression (RT-PCR, normalized to *β-actin*). Data is presented as mean ± SD or median (interquartile range); ^*∗∗*^*P* < 0.01 and ^*∗*^*P* < 0.05.

**Figure 9:** The RC decoction effects on the ALI and NETs under the CXCR2 expression suppression. (a) Lung wet weight/body weight ratio (LW/BW). (b) Lung HE staining (200x magnification, bar = 50 *μ*m) and lung injury scores. (c) The blood neutrophil (NEU) percent (flow cytometry). (d) Plasma NE-DNA relative concentration (ELISA). (e) Lung tissues NETs formations detected by the immunofluorescence (left, bar = 50 *μ*m; red: cit-H3, green: myeloperoxidase, blue: DNA), with the colocalization quantitative analyses (right). Data is presented as mean ± SD or median (interquartile range); ^*∗*^*P* < 0.05.

**Table 1:** Summary of the Renshen and Chishao active compounds.

Herb	Compound Id	Molecule name	OB (%)	DL
Chishao	MOL000359	Sitosterol	36.91	0.75
Chishao	MOL000492	(+)-catechin	54.83	0.24
Chishao	MOL001002	Ellagic acid	43.06	0.43
Chishao	MOL001918	Paeoniflorgenone	87.59	0.37
Chishao	MOL001921	Lactiflorin	49.12	0.80
Chishao	MOL001924	Paeoniflorin	53.87	0.79
Chishao	MOL001925	paeoniflorin_qt	68.18	0.40
Chishao	MOL002714	Baicalein	33.52	0.21
Chishao	MOL002776	Baicalin	40.12	0.75
Chishao	MOL002883	Ethyl oleate (NF)	32.40	0.19
Chishao	MOL004355	Spinasterol	42.98	0.76
Chishao	MOL005043	Campest-5-en-3beta-ol	37.58	0.71
Chishao	MOL006990	(1S,2S,4R)-trans-2-hydroxy-1,8-cineole-B-D-glucopyranoside	30.25	0.27
Chishao	MOL006992	(2R,3R)-4-methoxyl-distylin	59.98	0.30
Chishao	MOL006994	1-o-Beta-d-glucopyranosyl-8-o-benzoylpaeonisuffrone_qt	36.01	0.30
Chishao	MOL006996	1-o-Beta-d-glucopyranosylpaeonisuffrone_qt	65.08	0.35
Chishao	MOL006999	Stigmast-7-en-3-ol	37.42	0.75
Chishao	MOL007003	Benzoyl paeoniflorin	31.14	0.54
Chishao	MOL007004	Albiflorin	30.25	0.77
Chishao	MOL007005	Albiflorin_qt	48.70	0.33
Chishao	MOL007008	4-Ethyl-paeoniflorin_qt	56.87	0.44
Chishao	MOL007012	4-o-Methyl-paeoniflorin_qt	56.70	0.43
Chishao	MOL007014	8-Debenzoylpaeonidanin	31.74	0.45
Chishao	MOL007016	Paeoniflorigenone	65.33	0.37
Chishao	MOL007018	9-Ethyl-neo-paeoniaflorin A_qt	64.42	0.30
Chishao	MOL007022	Evofolin B	64.74	0.22
Chishao	MOL007025	Isobenzoylpaeoniflorin	31.14	0.54
Chishao, Renshen	MOL000358	Beta-sitosterol	36.91	0.75
Chishao, Renshen	MOL000449	Stigmasterol	43.83	0.76
Renshen	MOL000422	Kaempferol	41.88	0.24
Renshen	MOL000787	Fumarine	59.26	0.83
Renshen	MOL002879	Diop	43.59	0.39
Renshen	MOL003648	Inermin	65.83	0.54
Renshen	MOL004492	Chrysanthemaxanthin	38.72	0.58
Renshen	MOL005308	Aposiopolamine	66.65	0.22
Renshen	MOL005314	Celabenzine	101.88	0.49
Renshen	MOL005317	Deoxyharringtonine	39.27	0.81
Renshen	MOL005318	Dianthramine	40.45	0.20
Renshen	MOL005320	Arachidonate	45.57	0.20
Renshen	MOL005321	Frutinone A	65.90	0.34
Renshen	MOL005344	Ginsenoside rh2	36.32	0.56
Renshen	MOL005348	Ginsenoside-Rh4_qt	31.11	0.78
Renshen	MOL005356	Girinimbine	61.22	0.31
Renshen	MOL005357	Gomisin B	31.99	0.83
Renshen	MOL005360	Malkangunin	57.71	0.63
Renshen	MOL005376	Panaxadiol	33.09	0.79
Renshen	MOL005384	Suchilactone	57.52	0.56
Renshen	MOL005399	alexandrin_qt	36.91	0.75
Renshen	MOL005401	Ginsenoside Rg5_qt	39.56	0.79

## Data Availability

The data underlying this article will be shared upon reasonable request to the corresponding author.
